This article has been retracted.

# Design of Intelligent Nursing Decision Support System Based on Multiattribute Decision Model

**DOI:** 10.1155/2022/1088393

**Published:** 2022-01-28

**Authors:** Wenjing Lu, Wei Jiang, Na Zhang, Feng Xue

**Affiliations:** Nursing Department, The Second Affiliated Hospital of Air Force Military Medical University, Xi'an 710038, China

## Abstract

Nursing medical histories are copied randomly, leading to the occurrence of incorrectly altered histories, and medical errors are on the rise year by year. Moreover, erroneous falsification of nursing medical history is a challenging issue that needs to be urgently addressed in domestic nursing medical history. In this manuscript, a caregiver association method, which is based on a multiattribute decision model, is proposed which is specifically designed for the caregiver association selection problem in intelligent caregiving decision making. In this mode, through the selection and modeling of key performance indicators and the design of combined weights, the purpose of regulating the priority of attributes is achieved. At the same time, a comprehensive evaluation index is designed to realize the joint optimization of multiple attributes. Simulation results show that the proposed nursing workstation can not only tradeoff the quality of nursing staff experience and system performance but also balance the distribution of nursing work and effectively reduce the association delay and system energy consumption．

## 1. Introduction

Medical record is a record of medical activities formed by medical personnel after obtaining relevant information through consultation, physical examination, auxiliary examination, diagnosis, treatment, nursing, and other medical activities, and then summarizing, analyzing, and organizing these in a documented form [1–5]. Likewise, nursing assessment is a systematic, purposeful, and planned process of collecting information about a patient's condition while in the hospital. Based on the information collected about the patient's condition, a general nursing assessment is made about the subject of care and the surrounding area, which provides the basic basis for nursing activities. The nursing assessment is the foundation of the entire nursing process and is the most central step in the implementation of nursing activities. Inaccurate estimates can lead to errors in nursing diagnosis and care planning, as well as a failure of desired goals. The nursing assessment decision support system (NADSS) evolved from the development of the traditional nursing assessment, which contains all information from all paper assessment sheets, i.e., all original records of the patient's entire care process during the hospital stay. The American Academy of Nursing recommends the inclusion of standard nursing language in modern electronic health records (EHRs) to standardize nursing data and support clinical nursing practice [6–8].

The nursing assessment instrument contains an admission assessment form, an admission notification form, an in-hospital assessment form, an inpatient nursing record, an inpatient nursing record, and a perioperative nursing assessment. The perioperative nursing assessment is further subdivided into preoperative preparation assessment (preoperative day), preoperative preparation assessment (preoperative evening), preoperative day preoperative assessment, assessment at admission to the operating room, intraoperative assessment and care, postoperative assessment in the operating room, postoperative day postoperative assessment (ward), and surgical nursing assessment. Each nursing assessment consists of two parts: the patient's hospitalization information and the nursing assessment instrument. As the main body of the nursing assessment, it contains the assessment of living habits and self-care, physiological status, nutritional status, mucosal and skin condition, respiratory system, circulatory system, digestive and urinary system, pain and mental health, cannulation status, and specialty assessment. Each section is made up of paragraphs, which in turn are made up of medical elements.

In this manuscript, a caregiver association method, which is based on a multiattribute decision model, is proposed which is specifically designed for the caregiver association selection problem in intelligent caregiving decision making. In this mode, through the selection and modeling of key performance indicators and the design of combined weights, the purpose of regulating the priority of attributes is achieved. At the same time, a comprehensive evaluation index is designed to realize the joint optimization of multiple attributes. The subsequent sections of this paper are arranged according to the following agenda items.

In Section 2, related work is thoroughly analyzed with strong emphasis on the identification of issues in various methods.

## 2. Related Work

The concept of nursing assessment was first introduced in the United States by Pesut and Herman, and their findings are based on the development of the U.S. health delivery system. They have observed that the nursing process would evolve through six phases from its emergence in 1950 to 2050. (i) Phase 1 (1950–1969) focused on nursing problem solving and emphasized nursing assessment (nursing diagnosis was the conclusion of nursing assessment). (ii) Phase 2 (1970–1989) focused on nursing diagnosis and diagnostic reasoning. (iii) Phase 3 (1990–2009) focused on the development of a conjuncture-oriented model supported by the four judgmental line and clinical reasoning. (iv) Phase 4 (2010–2024) analyzes the models and relationships among nursing diagnoses, nursing measures, and nursing angles, and refines these values. (v) Phase 5 (2025–2034) is the establishment of a nursing prototype based on experience and justification. (vi) Phase 6 (2035–2050) is the development of forward-looking nursing based on the nursing prototype [8–12].

The above is a strategic plan for nursing assessment made by the U.S. health delivery system, developed at each different time to incorporate specific contexts and needs. Countries around the world are now developing their own nursing disciplines, using the United States as a model. As you can see from the plan, the U.S. is in Stage 4, which means that it has basically completed the collection of big data on basic nursing information and the construction of nursing models, and is moving toward standardized clinical good to support decision making.

In brief summary, the directions for the development of clinical decision systems for nursing assessment abroad are listed below:

1. Standardization of the nursing assessment process
2. The use of standard nursing language
3. Inclusion of nursing diagnosis
4. Computerized nursing support systems
5. Outcome-oriented models
6. Forward-looking clinical nursing-assisted decision making

China introduced nursing procedures from abroad in the early 1980s, and the nursing procedures proposed by the American Academy of Nursing have been the basic working methods recognized by nursing in Chinese health institutions. However, compared to foreign countries, hospital informatization in China started late and has a weaker foundation. Although after more than 30 years of independent development and the state has invested a lot of human and financial resources, there are still a large number of difficulties and deficiencies in the complex environment of hospitals, and the level of nursing assessment applications is still at the primary stage of development, a large part of which is due to the lack of various standards and relevant laws in the medical field [13–15].

The assessment phase is the stage that provides a solid foundation for implementing high-quality individualized care, but in clinical practice, the patient assessment process is often only formal and does not truly and objectively reflect the patient's health problems due to factors such as the nurse's own quality and the current state of nursing care. The main deficiencies include the following:

1. Most hospitals will develop nursing assessment sheets, but the content is not detailed enough, only simply recording the patient's vital signs, cultural background, personality habits, health status, and self-care ability, but failing to assess the physiological status of the patient's systems, making the quality of care not indepth and sustainable
2. A few hospitals have also established assessment sheets according to the system, but they fail to achieve screening and early warning functions for high-risk groups, making the nursing assessment serve only a simple function of recording patient information
3. No hospital has yet reported the ability to objectively and automatically generate a graded care level for the day based on the content of patient care assessment information, making the determination of graded care levels in most hospitals somewhat arbitrary
4. Most hospitals also have inconsistent physician-nurse records due to inconsistencies in the level of expertise and judgment of medical conditions between physicians and nurses, which is the key legal problem of poor proof in the event of a potential medical malpractice dispute

China's Ministry of Health issued the “Basic Standards for Medical Record Writing (Trial)” in 2002, followed by the “Basic Standards for Medical Record Writing” on January 22, 2010, and created the necessary legal, ethical, and policy structures to drive the development of nursing assessment by establishing a medico-legal working group to explore medico-legal issues such as the privacy and confidentiality of patients' health information and mature environmental conditions.

However, on the one hand, because nursing assessment involves all aspects of hospital informatization and is highly coupled and complex, more than 40% of medical institutions nationwide still use the traditional paper-based nursing chart writing mode or simply replace the pen with a computer to write nursing charts. As a result, most of the nursing medical record data cannot be explored in depth, and a mountain of precious clinical nursing data is wasted in this way.

On the other hand, there is no same set of norms for nursing assessment in the actual use process, and nurses are more arbitrary in writing medical records, which leads to the low quality of nursing medical records, and the supervisory department is unable to carry out unified and effective informational supervision. Nursing medical histories are copied randomly, leading to the occurrence of incorrectly altered histories, and medical errors are on the rise year by year. Erroneous falsification of nursing medical history is also an important issue that needs to be urgently addressed in domestic nursing medical history at present.

## 3. A Multiattribute Decision Model Based on Caregiver Association Algorithm

In this section, a multiattribute enabled decision model which is primarily based on the caregiver association algorithm is presented along with a comprehensive discussion and explanation.

### 3.1. A Model for the Caregiver Association Multiattribute Decision Problem

#### 3.1.1. Associated Decision Makers and Decision Care Workstations

Caregiver *u*_*i*_ needs to select the appropriate care workstation for association in the set F of care workstations to be selected so that caregiver *u*_*i*_ is the decision maker, and the *L* care workstations to be selected are the alternative care workstations, i.e., the associated decision care workstations.

#### 3.1.2. Associated Decision Attribute Set

In addition to retaining the reference signal receiving power (RSRP), which is considered by the traditional association algorithm, six KPIs, namely task processing delay, system energy consumption, caregiver payment cost, remaining communication capacity of the caregiver workstation, and remaining computational capacity of the caregiver workstation are selected to construct the caregiver association decision attribute set. Among them, three attributes, RSRP, task processing delay, and caregiver payment cost, are used to measure the caregiver QoE under the proposed scenario model, and the remaining three attributes are used to measure the performance of the system. Among the six KPIs, RSRP, remaining communication capacity of the nursing workstation, and computational capacity are physical quantities that characterize the resource intensity of the nursing workstation without complex modeling design and are denoted by *C*^ref ^, *C*^*trans*_*r*_*est*^, and *C*^exe_rest ^, respectively, and the specific values are randomly generated within the range of value set by the simulation.

#### 3.1.3. Associative Decision Matrix and Normalization

Assume that the set of attributes of the nursing workstations in the network contains a total of *M* attributes. Corresponding the *L* nursing workstations to be selected by the nursing staff *u*_*i*_ to the row vectors of the decision matrix and the attribute values of the *M* attributes to the column vectors of the matrix, the nursing staff association decision matrix *A*_*L*×*M*_ is

(1) $$\begin{array}{c} A_{L\times M}=\left[\begin{array}{cccc} a_{11} & a_{12} & \cdots & a_{1M}\\ a_{21} & a_{22} & \cdots & a_{2M}\\ \vdots & \vdots & \vdots \\ a_{L1} & a_{L2} & \cdots & a_{LM} \end{array}\right], \end{array}$$

where element *a*_*ml*_(*l*=1,2,…, *L*; *m*=1,2,…, *M*) is the m*th* attribute value of the l*th* nursing workstation in the set F of nursing workstations to be selected.

The normalization of the attribute values using the polar transformation method consists of the following 3 steps．

**Step 1 .**

Among the six selected attributes, RSRP, the remaining communication capacity of the nursing workstation, and the remaining computational capacity of the nursing workstation are benefit-based attributes. The benefit-based attributes are normalized according to the following equation:

(2) $$\begin{array}{c} r_{lm}^{+}=\frac{a_{lm}-\min_{l}a_{lm}}{\max_{l}a_{lm}-\min_{l}a_{lm}}, \end{array}$$

**Step 2 .**

Inversely with the benefit-type property, the cost type is normalized by equation (2).

(3) $$\begin{array}{c} r_{lm}^{-}=\frac{\max_{l}a_{lm}-a_{lm}}{\max_{l}a_{lm}-\min_{l}a_{lm}}, \end{array}$$

where min_*l*_*a*_*lm*_ is the smallest attribute in column *m* of *A*_*L*×*M*_, and max_*l*_*a*_*lm*_ is the largest attribute in column *m* of *A*_*L*×*M*_.

**Step 3 .**

The normalized correlation decision matrix is obtained after the attribute normalization process as

(4) $$\begin{array}{c} R_{L\times M}=\left[\begin{array}{cccc} r_{11} & r_{12} & \cdots & r_{1M}\\ r_{21} & r_{22} & \cdots & r_{2M}\\ \vdots & \vdots & \vdots \\ r_{L1} & r_{L2} & \cdots & r_{LM} \end{array}\right], \end{array}$$

where element *r*_*lm*_ is the value of each attribute after normalization.

#### 3.1.4. Portfolio Weighting Design

**Step 4 .**

Subjective weight acquisition. The subjective weights are determined by subjective factors such as nursing staff preferences and the use of computing resources at the nursing workstation. The subjective weight value of each attribute is expressed as *ω*_*m*_^*s*^ , which forms the subjective weight vector *ω*^*s*^ with

(5) $$\begin{array}{c} \omega^{s}={\left[\omega_{1}^{s},\cdots ,\omega_{m}^{s},\cdots ,\omega_{M}^{s}\right]}^{T}, \end{array}$$

where the superscript *s* is the subjective identifier of the subjective weight, and *m* is the index of the m*th* weight value element in the weight vector *ω*^*s*^.

**Step 5 .**

The objective weights of the attributes are obtained using the entropy weight method. The objective weight vector is denoted as *ω*^*o*^=[*ω*_1_^*o*^, ⋯,*ω*_*m*_^*o*^, ⋯,*ω*_*M*_^*o*^]^*T*^. The application of the entropy weight method to determine the objective weights *ω*_*m*_^*o*^ consists of 2 steps.

First, the entropy value *e*_*m*_ of the m*th* attribute is expressed as

(6) $$\begin{array}{c} e_{m}=-\ln\;{\left(L\right)}^{-1}\sum_{l=1}^{L}p_{lm}\ln\;p_{lm}, \end{array}$$

where *p*_*lm*_=*r*_*lm*_/∑_*l*=1_^*L*^*r*_*lm*_;

second, based on the entropy value *e*_*m*_, the objective weight of the m*th* attribute is

(7) $$\begin{array}{c} \omega_{m}^{o}=\frac{1-e_{m}}{\sum_{m=1}^{M}\left(1-e_{m}\right)}. \end{array}$$

**Step 6 .**

The combination weights are determined. Based on the principle of minimum discriminative information, the objective function for solving the combined weight value *ω*_*m*_ is constructed as

(8) $$\begin{array}{c} \min_{\omega_{m}}F=\min_{\omega_{m}}\left\{\sum_{m=1}^{M}\omega_{m}\left(\ln\frac{\omega_{m}}{\omega_{m}^{s}}\right)+\sum_{m=1}^{M}\omega_{m}\left(\ln\frac{\omega_{m}}{\omega_{m}^{{}^{\circ}}}\right)\right\},\\ s.t.\;C1:\overset{M}{\underset{m=1}{\sum }}\omega_{m}=1C2:\omega_{m}>0, \end{array}$$

where *ω*_*m*_ is the combination weight of the m*th* attribute of the associated care workstation; the constraint C1 is the sum of the combination weights of all attributes corresponding to 1, and C2 is the non-negative weight of each combination. A Lagrangian function is constructed with respect to the objective function with respect to *ω*_*m*_; it is denoted as

(9) $$\begin{array}{c} L\left(\omega_{m},\xi_{1},\xi_{2}\right)=\overset{M}{\underset{m=1}{\sum }}\omega_{m}\left(2\;\ln\;\omega_{m}-\ln\;\omega_{m}^{0}\omega_{m}^{\text{s}}\right)\\ +\xi_{1}\left(\overset{M}{\underset{m=1}{\sum }}\omega_{m}-1\right)+\xi_{2}\left(-\omega_{m}\right), \end{array}$$

where *ξ*_1_ and *ξ*_2_ are the Lagrangian multipliers corresponding to constraints C1 and C2, respectively. The Lagrangian function is solved to obtain the combined weights with

(10) $$\begin{array}{c} \omega_{m}=\frac{{\left(\omega_{m}^{s}\omega_{m}^{o}\right)}^{1/2}}{\sum_{m=1}^{M}{\left(\omega_{m}^{s}\omega_{m}^{0}\right)}^{1/2}}. \end{array}$$

#### 3.1.5. Decision Matrix Weighting

The weighted normalized decision matrix *U*_*L*×*M*_=[*u*_*lm*_]_*L*×*M*_=[*ω*_*m*_*r*_*lm*_]_*L*×*M*_ is obtained by multiplying the attribute values *r*_*lm*_ in the normalized correlation decision matrix *R*_*L*×*M*_ with their corresponding combined weight values *ω*_*m*_ , i.e.,

(11) $$\begin{array}{c} U_{L\times M}=\left[\begin{array}{cccc} u_{11} & u_{12} & \cdots & u_{1M}\\ u_{21} & u_{22} & \cdots & u_{2M}\\ \vdots & \vdots & \vdots \\ u_{L1} & u_{L2} & \cdots & u_{LM} \end{array}\right], \end{array}$$

where element *u*_*lm*_ is the weighted normalized value of each attribute.

### 3.2. Best Associated Care Workstation

Considering the superiority-disadvantage solution distance method and the gray correlation analysis method, based on the above multiattribute decision model related design for the nursing staff association problem, the relative fit *l* for evaluating the superiority of the nursing workstation to be selected is constructed, and the steps are as follows:

**Step 7 .**

Determine the positive and negative ideal solutions for all associated nursing workstations. The positive ideal solution is the envisioned optimal nursing workstation [16–20], and the negative ideal solution is the envisioned worst nursing workstation. The number of attributes selected is *M* = 6. Assuming that the control unit constructs the attribute set by assigning 3 benefit attributes to the first 3 columns of the decision matrix and the remaining 3 cost attributes to the last 3 columns, the positive ideal solution **u**^+^ and the negative ideal solution **u**^−^ for the nursing staff-associated nursing workstations are

(12) $$\begin{array}{c} u^{+}=\left[\max_{1\leq l\leq L}u_{l1},\max_{1\leq l\leq L}u_{l2},\max_{1\leq l\leq L}u_{l3},\min_{1\leq l\leq L}u_{l4},\min_{1\leq l\leq L}u_{l5},\min_{1\leq l\leq L}u_{l6}\right],\\ u^{-}=\left(21\right)\left[\min_{1\leq l\leq L}u_{l1},\min_{1\leq l\leq L}u_{l2},\min_{1\leq l\leq L}u_{l3},\max_{1\leq l\leq L}u_{l4},\max_{1\leq l\leq L}u_{l5},\max_{1\leq l\leq L}u_{l6}\right]. \end{array}$$

**Step 8 .**

Calculate the Euclidean between each associated care workstation and the ideal solution

Distance. The Euclidean distances of the l*th* associated care workstation **u**_*l*_=[*u*_*l*1_, *u*_*l*2_,…, *u*_*l*6_] in **U**_*L*×*M*_ from the positive ideal solution **u**^+^ and the negative ideal solution **u**^−^ are

(13) $$\begin{array}{c} D_{l}^{+}={\left\|u_{l}-u^{+}\right\|}_{2},\\ D_{l}^{-}={\left\|u_{l}-u^{-}\right\|}_{2}. \end{array}$$

**Step 9 .**

Calculate the gray correlation between each associated care station and the ideal solution. First, the gray correlation coefficients *g*_*lm*_^+^ and *g*_*lm*_^−^ between **u**_*l*_ and the positive ideal solution **u**^+^ and the negative ideal solution **u**^−^ with respect to the m*th* attribute are

(14) $$\begin{array}{c} g_{lm}^{+}=\frac{\min\min_{l}\left|u_{m}^{+}-u_{lm}\right|+\eta \max\max_{l}\left|u_{m}^{+}-u_{lm}\right|}{\left|u_{m}^{+}-u_{lm}\right|+\eta \max_{l}\max_{m}\left|u_{m}^{+}-u_{lm}\right|},\\ g_{lm}^{-}=\frac{\min_{l}\min_{m}\left|u_{m}^{-}-u_{lm}\right|+\eta \max\max_{l}\left|u_{m}^{-}-u_{lm}\right|}{\left|u_{m}^{-}-u_{lm}\right|+\eta \max_{l}\max_{m}\left|u_{m}^{-}-u_{lm}\right|}, \end{array}$$

where *u*_*m*_^+^ and *u*_*m*_^−^ are the elemental values of the m*th* attribute in the positive ideal solution **u**^+^ and the negative ideal solution **u**^−^, respectively, **u**_*lm*_ is the elemental value of the m*th* attribute of the l*th* associated care workstation **u**_*l*_, and *η* is the discrimination coefficient, which takes the value of 0 < *η* < 1 and is usually taken as 0.5 based on experience [21–24].

Second, the gray correlation coefficients *g*_*l*_^+^ and *g*_*l*_^−^ of *u*_*l*_ with the positive ideal solution *u*^+^ and the negative ideal solution, respectively, are

(15) $$\begin{array}{c} g_{l}^{+}=\frac{1}{M}\overset{M}{\underset{m=1}{\sum }}g_{lm}^{+},\\ g_{l}^{-}=\frac{1}{M}\overset{M}{\underset{m=1}{\sum }}g_{lm}^{-}. \end{array}$$

**Step 10 .**

Construct the relative fit for evaluating the strengths and weaknesses of the associated nursing workstation. First, the Euclidean distance and the gray correlation degree are normalized by the measure according to the following equation:

(16) $$\begin{array}{c} \alpha_{l}^{\prime }=\frac{\alpha_{l}}{\max_{1\leq l\leq L}\alpha_{l}}, \end{array}$$

where *α*_*l*_ can be substituted into *D*_*l*_^+^, *D*_*l*_^−^, *g*_*l*_^+^, and *g*_*l*_^−^, respectively.

Second, the positive and negative judgment indicators of the combined two are defined as

(17) $$\begin{array}{c} Q_{l}^{+}=\xi D_{l}^{-}+\left(1-\xi \right)g_{l}^{+},\\ Q_{l}^{-}=\xi D_{l}^{+}+\left(1-\xi \right)g_{l}^{-}, \end{array}$$

where *ξ* is the preference parameter．

Finally, the relative fit was constructed based on *Q*_*l*_^+^ and *Q*_*l*_^−^:

(18) $$\begin{array}{c} l=\frac{Q_{l}^{+}}{Q_{l}^{+}+Q_{l}^{-}}. \end{array}$$

The largest nursing workstation in the nursing workstation association decision matrix is the best associated nursing workstation for the nursing staff to choose．

### 3.3. A Multiattribute Decision Model Based Caregiver Association Algorithm

**Step 11 .**

The nursing workstation receives the association decision request from the nursing staff, calculates and generates *M* attribute values of all nursing workstations in the network using the attribute-related information collected by the control unit in advance, and selects the nursing workstations satisfying the capacity and time delay constraints from all nursing workstations according to equation (18) to construct the nursing workstation association decision set *F*={*f*_1_, *f*_2_,…, *f*_*L*_}.

(19) $$\begin{array}{c} \varepsilon_{i}\leq C_{j}^{texe_{r}est}\\ d_{i}\leq C_{j}^{trans_{r}est}\\ T_{j,i}^{all}\leq T_{i}^{\max}, \end{array}$$

where *C*_*j*_^t*exe*_*r*_*est*^ is the remaining computational capacity of the nursing workstation *k*_*j*_(*k*_*j*_ ∈ Φ); *C*_*j*_^*trans*_*r*_*est*^ is the remaining communication capacity of the nursing workstation *k*_*j*_; *T*_*j*,*i*_^all^ is the latency corresponding to the association of the nursing staff *u*_*i*_ with the nursing workstation *k*_*j*_; and *T*_*i*_^max^ is the maximum latency that can be tolerated for the computational tasks of the nursing staff *u*_*i*_.

**Step 12 .**

Calculate the association decision matrix *A*_*L*×*M*_ using equation (10), normalize each attribute value in *A*_*L*×*M*_ according to equation (11) and equation (12), and generate the normalized association decision matrix *A*_*L*×*M*_ by equation (14).

**Step 13 .**

Calculate the combination weights corresponding to each attribute value *r*_*lm*_ in *R*_*L*×*M*_ based on equations. (15), (17), and (19) with respect to *ω*_*m*_.

**Step 14 .**

Calculate the weighted normalized decision matrix after the attribute values *r*_*lm*_ are weighted by *ω*_*m*_ using equation (19).

**Step 15 .**

Calculate the gray correlation between each associated nursing workstation and the positive and negative ideal solutions by calculating the Euclidean distance between each associated nursing workstation and the positive and negative ideal solutions using equation (19).

**Step 16 .**

Normalize *D*_*l*_^+^, *D*_*l*_^−^, *g*_*l*_^+^, and *g*_*l*_^−^ according to equation (19) and calculate the positive and negative judgments of the combined Euclidean distance and gray correlation indexes *Q*_*l*_^+^ and *Q*_*l*_^−^.

**Step 17 .**

By calculating the final judgment index *l* for evaluating the merit of the associated nursing workstation and using equation (18) to select the index *l*^*∗*^ of the best performing nursing workstation, the nursing workstation feeds this result to the nursing staff, who selects the nursing workstation *f*_*l*^*∗*^_ for association.

(20) $$\begin{array}{c} l^{*}=\underset{l\in \left\{1,2,3,\ldots ,L\right\}}{\arg\min}\left(L\right). \end{array}$$

## 4. Simulation Result and Analysis

### 4.1. Parameter Setting

Simulation scenario consists of 3 patients with severe illness and 6 patients with light illness. The coverage radius of the nursing workstation is set to 500 m and 50 m, and the three nursing workstations are placed at three vertices in a square area with 800 *m* × 800 m sides, while each of the six nursing workstations is randomly distributed in the simulation area of its own nursing workstation according to the chi-square Poisson point process, and the nursing staff are evenly distributed in the coverage area of the nursing workstation. All simulation results are taken from the average of 1,200 independent simulations．

### 4.2. Simulation Performance Analysis

To facilitate the comparison and analysis of simulation results, the following three nursing workstations are set up. The nursing workstation 1 proposes a multiattribute decision model-based nursing staff association algorithm. The nursing workstation 2 proposes a coefficient adjustable Hungarian algorithm-based nursing staff association nursing workstation, which optimizes the goal of communication load balancing [6]. The delay minimization nursing staff association algorithm is proposed in nursing workstation 3 [7].  Figure 1 shows the cumulative distribution of the time delay probability of a single caregiver with the number of caregivers being 100 and the subjective weight vector *ω*_*s*_ set to [0.1, 0.1, 0.1, 0.4, 0.2, 0.1] *T* for different coverage of the sickest patients. The subjective weight value of the time delay is 0.4. As seen in Figure 1, the single caregiver time delay of the proposed algorithm is lower than that of the other 2 caregiver workstations within any severely ill patient．

Figure 2 shows the relationship between the total energy consumption of the system and the number of nursing staff in the network for *ω*_*s*_ settings of [0.15, 0.1, 0.1, 0.1, 0.4, 0.15] T. The subjective weight value of energy consumption is set to 0.4. As seen in Figure 2, the proposed nursing workstation has the lowest energy consumption with a different number of nursing staff, and the trend of energy consumption increases more slowly. This is because the proposed nursing workstation can directly optimize the energy consumption by making the energy consumption of the system one of the cost-based attributes of the correlation decision, which makes the energy consumption one of the optimization objectives of the correlation decision.

Figure 3 shows the comparison of communication load and computational load of six nursing workstations selected from three coverage areas of very sick patients when the number of nursing staff is 100 and *ω*_*s*_ is set to [0.1, 0.1, 0.1, 0.4, 0.25, 0.05] T. Among these, subjective weight values of the remaining computational capacity and the remaining communication capacity are set to 0.1. As seen in Figure 3, the proposed nursing workstations are most effective in optimizing the degree of patient care.

Figure 4 shows the average delay and total system energy consumption of the proposed algorithm as a function of the number of nursing staff for different genders of the nursing workstation scores, respectively. As can be seen, both the average delay and the system energy consumption decrease with increasing subjective weights of the corresponding delay and energy consumption for any number of caregivers. Although the variation of only two of the six attributes selected for Care Workstation 1 is evaluated, it is sufficient to show that the proposed algorithm can control the priority of each attribute by controlling the subjective weight value of each attribute, thus achieving a tradeoff between caregivers and system performance.

In addition, the predicted patient degree of care data from the 10 groups was brought into the model to derive the corresponding patient degree of care type, which was verified by comparison with the actual condition. In order to verify the true accuracy, this subsection was tested based on this patient care degree data classification, thus diagnosing the degree of patient care based on this model for the turnout, as shown in Figures 5 and 6. After system testing, the results achieved 100% correctness, and unreliability was only 0%. The experiments showed that this model has a good capability of patient care degree, which can be intelligently diagnosed by the complexity analysis created by the algorithm. The analysis from the perspective of patient care participation based on the degree of patient care shows that the intelligent diagnosis of the degree of patient care is superior to the intelligent patient care degree diagnosis based on the traditional degree of patient care.

## 5. Conclusion and Future Directions

In this paper, we have proposed a nursing staff association method, which was based on a multiattribute decision model. In the proposed model, we have used selection and modeling of key performance indicators along with the design of combination weights to successfully achieve the expected level of performance, which was the ultimate purpose of regulating the priority of attributes. At the same time, a comprehensive evaluation index is designed to realize the joint optimization of multiple attributes. Simulation results show that the proposed nursing workstation can not only tradeoff the quality of nursing staff experience and system performance but also balance the distribution of nursing work.

In the future, we are eager to apply and implement the proposed mechanism in a real working environment of smart Internet of Things-enabled hospital management system.

## Figures and Tables

**Figure 1:** Cumulative distribution of probability of time delay for a single caregiver.

**Figure 2:** Relationship between nursing staff work status and number of patients.

**Figure 3:** Work intensity of nurses.

**Figure 4:** Scores of different nursing workstations.

**Figure 5:** Operating error of different nurses.

**Figure 6:** Level of care for different patients.

## Data Availability

The datasets used and analyzed during the current study are available from the corresponding author upon reasonable request.
